This article has been retracted.

# Study on the Relationship between Different Body Mass Indexes and Puncture Pain and Image Quality in Patients Undergoing Coronary Angiography with Intravenous Indwelling Needle

**DOI:** 10.1155/2022/4105875

**Published:** 2022-05-19

**Authors:** Jiani Ding, Xiaoyu Chen

**Affiliations:** ^1^Department of Outpatient Service, The First Affiliated Hospital of Wenzhou Medical University, Wenzhou 325005, Zhejiang, China; ^2^Department of Radiology, The First Affiliated Hospital of Wenzhou Medical University, Wenzhou 325005, Zhejiang, China

## Abstract

**Objective:**

To investigate the effect of different body mass indexes (BMIs) on patients' puncture pain, puncture success rate, and image quality in coronary angiography (CAG) performed with an intravenous indwelling needle, and to provide a basis for selecting the appropriate intravenous indwelling needle for CAG in patients with different BMIs in an outpatient clinic.

**Method:**

In this study, 300 patients undergoing CTA at the department of radiology in the First Affiliated Hospital of Wenzhou Medical University from January to May 2021 were divided into group 1 (BMI 1 ≤ 18.5), group 2 (18.5 < BMI ≤ 24), and group 3 (BMI > 24) according to their BMI, with 100 cases in each group, and a 20 G intravenous indwelling needle was used in each group. The age, sex, height, and weight of each patient were recorded, and the primary puncture success rate, contrast leakage rate, injection success rate, pain perception, and subjective ratings of image quality and objective indicators were compared in patients with different BMI values.

**Results:**

There was no statistically significant difference between the age, gender, and heart rate of the patients in the three groups (*P* > 0.05). There was no statistically significant difference between the primary puncture success rate, injection success rate, and contrast leakage rate of the three groups of patients (*P* > 0.05). The pain scores of group 3 during contrast injection were significantly higher than those of the remaining two groups (*P* < 0.05), while the differences between the pain scores of group 2 and group 1 during contrast injection were not statistically significant (*P* > 0.05); the comparison of the pain scores of the three groups during puncture and during retention was not statistically significant (*P* > 0.05). The differences between the subjective ratings of image quality and the objective indicators of the three groups were not statistically significant (*P* > 0.05).

**Conclusion:**

The 20 G indwelling needle can basically meet the coronary angiography examination of patients with different body mass indexes, but patients with a BMI greater than 24 are recommended to use a larger diameter indwelling needle to reduce contrast leakage as well as to reduce patient pain and improve patient comfort.

## 1. Introduction

The incidence of coronary artery disease (CAD) is gradually on the rise as people's lifestyles change, making its early diagnosis and risk stratification increasingly important [1]. Currently, several tests including ECG, myocardial stress test, and CT angiography are helpful in the diagnosis of CAD [2]. Among them, CT angiography (CTA) has been increasingly used for the examination and diagnosis of the cardiovascular system due to its convenience and minimally invasive nature [3]. In CT scanning, when the density between the diseased tissue and normal tissue is relatively uniform, the contrast of the image formed after scanning is low, so that the diseased tissue is difficult to detect. There are many factors that influence the success or failure of coronary CTA examinations and the quality of imaging and analyzing the various influencing factors can help to provide a better development and application of this technique. Some studies [4, 5] have found that obesity is an independent and important risk factor for CAD and that weight is the most important influencing factor among patient factors affecting cardiac enhancement scans. The use of CT-enhanced scans can clearly distinguish the difference in uptake between diseased and normal tissues, and the successful completion of this method is closely related to the selection of different types of intravenous indwelling needles. In addition, the choice of indwelling needle type, although seemingly trivial, is related to the quality of coronary CTA image imaging and is therefore an issue that should not be ignored [6]. In order to obtain better enhancement, CTA imaging contrast injection is a high-dose, high-pressure, high-rate regimental injection, and the selection of the appropriate indwelling needle type is extremely important.

Therefore, this study was conducted to investigate the effects of using a 20 G intravenous indwelling needle on coronary CTA image quality and patient comfort in patients with different body mass indexes (BMIs), in order to provide references and suggestions for the selection of indwelling needle type for coronary CTA examination and better implementation of the coronary CTA technique.

## 2. Information and Methods

### 2.1. General Data

300 patients, aged 30–60 years, who underwent CTA in the outpatient clinic of the First Hospital of Wenzhou Medical University from October 2020 to May 2021 were selected, and their height and weight were recorded and BMI was calculated: BMI = weight (kg)/height (m^2^). The patients were divided into group 1 (BMI 1 ≤ 18.5), group 2 (18.5 < BMI ≤ 24), and group 3 (BMI > 24) according to BMI, with 100 cases in each group.

### 2.2. Consumables and Instruments

All the intravenous indwelling needles in this study were selected from the 20 G indwelling needles produced by Becton, Dickinson and Company in the United States. Philips 64-row spiral CT and Oulich high-pressure contrast injector pipeline system were used, and the contrast agent was 32% iontophoresis. The injection flow rate was 3–5 ml/s, and contrast agent injection dose was 1.4 ml/kg.

### 2.3. Method

According to the procedure of indwelling needle operation, a thick, straight, and flexible median elbow vein was selected, a tourniquet was tied about 5 cm above the puncture point after determining the puncture point, the skin was routinely disinfected twice with a disinfection range of >5 cm in diameter, and the needle was held with the skin at 15° to 30° into the needle. After seeing the blood return, lower the needle angle, continue to enter the needle 0.1–0.2 cm, then withdraw the needle core, and then send the outer casing into the vessel all in parallel, and again confirm the good blood return after fixing the indwelling needle with a disposable transparent dressing. Saline was finally aspirated with a 5 cm empty needle for intravenous push to prevent syringe reflux blockage.

After the patient entered the CT scan room, he or she was instructed to position himself or herself correctly, and the high-pressure syringe was mounted on the high-pressure syringe pump to draw the required amount of contrast medium. The catheter was connected and drained of air, the high-pressure syringe pump was placed in the appropriate position on the scan bed, and the heparin cap was removed and screwed to the catheter connector for backup. At the end of the leveling, the puncture site should be reconfirmed to be free of swelling before signaling the physician to activate the syringe pump switch. If swelling is found to be oozing, the injection should be stopped immediately and treated accordingly. If there was no swelling, the patient continued to be closely observed through the glass window for any adverse reactions until the end of the time-lapse scan. The needle was generally not usually removed urgently after the examination, but the intravenous needle was kept in place for 15 min so that this intravenous access could be used for rapid resuscitation in case of an allergic reaction.

### 2.4. Evaluation Methodology

#### 2.4.1. Successful Puncture

When puncture was performed, successful puncture was defined as the return of blood after venipuncture, smooth placement of the hose, and no swelling and nodules when saline was pushed. If there was no blood return, there was difficulty in sending the hose forward, or swelling and nodules would occur when saline was pushed in, and the patient complained of pain, the puncture failed.

*(1) Successful Injection*. When the contrast agent was pushed, the contrast agent was successfully injected into the patient with no swelling and oozing in and around the puncture site and no pain in the patient.

*(2) Contrast Agent Extravasation*. If the patient complains of obvious pain during injection and swelling at and around the puncture site, the contrast agent should be extravasated and the needle should be withdrawn immediately and treated accordingly.

#### 2.4.2. Image Quality Evaluation

The subjective rating was based on the American Heart Association coronary artery modified segmentation method with high quality: no artifacts and clear vessel boundaries. Good: mild artifacts or noise, which basically do not affect the evaluation. Barely diagnostic: severe motion artifacts or noise, but still able to evaluate the vascular lumen. Unable to evaluate or failed: severe artifacts or severe calcification were present, and the lumen could not be evaluated.

*(1) Objective Evaluation*. In cross section, CT values of aortic internal diameter (AO), proximal left anterior descending branch (LADp), distal left anterior descending branch (LADd), proximal right coronary artery (RCAp), distal right coronary artery (RCAd), proximal left circumflex branch (LCXp), and distal left circumflex branch (LCXd) were recorded in both groups, and the mean values were calculated and compared.

#### 2.4.3. Pain Scoring

The pain numerical scoring method was used to indicate the degree of pain by using the numerical formula 0–10 instead of words, and a straight line was divided into 10 equal segments to assess the degree of pain in the order of 0–10 points. The assessment was performed at the time of indwelling needle puncture and during indwelling and contrast injection, respectively.

### 2.5. Statistical Treatment

SPSS 19.0 statistical software was used for statistical processing, and Prism 8.0 was used for the production of statistical graphs. The measurement data were expressed as the mean ± standard deviation ($\bar{x}\pm s$), *t*/*F* test was used for comparison between groups, *χ*^2^ test was used for counting data, and *P* < 0.05 was considered statistically significant.

## 3. Results

### 3.1. Comparison of General Information of Patients in the Three Groups

There was no statistically significant difference between the three groups of patients in terms of age, gender, heart rate, clinical symptoms, and past medical history (*P* > 0.05) (Table 1).

### 3.2. Primary Puncture Success Rate, Injection Success Rate, and Contrast Leakage Rate in the Three Groups of Patients

There was no statistically significant difference between the primary puncture success rate, injection success rate, and contrast leakage rate in the three groups (*P* > 0.05) (Table 2).

### 3.3. Comparison of Pain Scores during Intravenous Needle Puncture, Retention, and Contrast Injection in the Three Groups

The differences in pain scores during intravenous needle puncture and retention were not statistically significant among the three groups (*P* > 0.05); during contrast injection, the pain scores in group 3 were significantly higher than those in groups 1 and 2 (*P* < 0.05), and the differences between groups 1 and 2 were not statistically significant (*P* > 0.05) (Figures 1(a)∼1(c)).

### 3.4. Comparison of Subjective Ratings of Image Quality among the Three Groups of Patients

There was no statistically significant difference in the comparison of the percentage of patients in the three groups with postexamination image quality ratings of good quality, good, barely diagnostic, and unable to assess/fail (*P* > 0.05) (Table 3).

### 3.5. Comparison of Objective Indicators of Image Quality among the Three Groups of Patients

There was no statistically significant difference (*P* > 0.05) in the comparison of CT values at the locations of AO (A), LADp (B), LADd (C), RCAp (D), RCAd (E), LCXp (F), and LCXd (G) among the three groups of patients (Figures 2(a)∼2(g)).

## 4. Discussion

CAD is among the most common types of cardiovascular diseases, and risk factors for CAD include hypertension, smoking, diabetes, physical inactivity, obesity, high blood cholesterol, depression, and alcohol overdose, and the underlying pathogenesis is due to cardiac atherosclerosis, which reduces blood flow as well as oxygen transfer to the myocardium [7, 8]. Epidemiological studies [9, 10] have shown that the number of overweight and obese people is increasing worldwide. The results of a cohort study [11] showed that an increase of 1 kg/m^2^ in BMI of study subjects stratified by BMI resulted in a 5–7% increase in the incidence of CAD and that obesity was an independent and important risk factor for CAD. CTA is a computed tomography technique that visualizes arterial and venous vessels throughout the body. This technique mainly involves the injection of contrast into the peripheral venous vessels, and when the contrast reaches the peak of filling in the peripheral vessels, a spiral CT is used to rapidly collect cross-sectional images to obtain validated raw images, and finally, the raw images are processed by computer to become three-dimensional images of the vessels [12, 13].

CTA has been widely used in the examination and diagnosis of coronary arteries. Coronary CTA requires a faster flow rate and a higher concentration of injectable contrast medium. The conventional scalp needle is a steel needle with a thick and sharp tip and a large bevel, which increases the chance of puncturing the vessel wall if the needle is too deep during the injection of the contrast agent, and if the needle is too shallow, it is easier to puncture the vessel wall due to the movement of the needle tip, in addition to the movement of the patient's body [14]. This can lead to leakage of the contrast agent. Since contrast agent is a hypertonic solvent, when the concentration is high, it is irritating to blood vessels and can easily cause damage to blood vessel walls and leakage, and extravasation of contrast agents can lead to tissue congestion and edema. Compared with ordinary steel needles, the IV indwelling catheter material is softer and less likely to pierce the vessel, which facilitates the smooth passage of the contrast medium and can reduce its extravasation to a certain extent [15]. Clinical studies [16] found that in coronary CTA examination, the injection flow rate of the injected contrast agent usually requires 5 mL/s. The relatively thin wall and large lumen of the intravenous indwelling needle significantly reduce the injection resistance during the injection process, ensuring the maximum injection flow rate making the contrast between the vessel and the surrounding tissue obvious and the vessel more visible and clear, thus improving the quality and effect of the scan image.

Although intravenous indwelling needles meet the needs of coronary CTA, the choice of different types of intravenous indwelling needles can have an impact on the outcomes of coronary angiography. A related study [17] found that the use of different types of indwelling needles for puncture resulted in different chances of contrast leakage and varying examination success and image quality. The study in [18] compared the effects of different types of indwelling needles in coronary vessels and found that the 18 G indwelling needle significantly improved the success rate of coronary angiography and reduced contrast leakage compared to the 24 G indwelling needle. However, the size of the indwelling needle is too small for contrast injection and CT examination, and the size of the indwelling needle is too large for the nurses to operate and increase the fear and pain of the patients, so it is important to choose the right size of the indwelling needle. One study [19] showed that among the patient factors affecting liver enhancement scans, weight is the most important one, as the high blood volume in obese patients leads to a more pronounced dilution of the contrast agent circulating in the body. Therefore, under the condition of fixing the total amount of contrast agent and injection rate, more contrast agent needs to be injected for high BMI to meet the clinical diagnostic requirements. However, BMI mainly reflects the fatness and body size characteristics of the patient, and an increase in weight is not linearly related to an increase in the contrast dose. To overcome the drawbacks of determining the contrast dose based solely on body weight, many studies have proposed to compare the amount of contrast agent used with net body weight and body surface area [20].

Therefore, in this paper, we used different BMI values of patients for group experiments and found that a 20 G indwelling needle can meet the examination needs of most patients, and the success rate of nurse operation is high and patient comfort is good. However, patients with higher BMI (especially >27) have increased contrast leakage and pain scores, and a larger size indwelling needle is recommended. In conclusion, there are many factors affecting the success of coronary CTA examination, including imaging quality and patient comfort, and the analysis of the various influencing factors can help to better develop and apply this technology. Therefore, choosing the appropriate needle placement type according to the patient's BMI size is beneficial to the contrast flow rate and group injection effect, which is important for improving the imaging quality of coronary CTA and patient comfort during the examination, and is worthy of clinical promotion.

## Figures and Tables

**Figure 1:** Comparison of pain scores among the three groups of patients (*n* = 100, $\bar{x}\pm s$, $\bar{x}$). Note: ^*∗*^group 1 compared with group 3, *P* < 0.05; #group 2 compared with group 1, *P* < 0.05. (a) The comparison of pain scores during puncture in the three groups; (b) the comparison of pain scores during retention in the three groups; (c) the comparison of pain scores during contrast injection in the three groups.

**Figure 2:** Comparison of objective indicators of image quality among the three groups of patients (*n* = 100, $\bar{x}\pm s$, $\bar{x}$). (a∼g) Comparison between the three groups of AO (a), LADp (b), LADd (c), RCAp (d), RCAd (e), LCXp (f), and LCXd (g), respectively.

**Table 1:** Comparison of age, sex, and heart rate among the three groups of patients (*n*, %; ($\bar{x}\pm s$)).

Information	Group 1 (*n* = 100)	Group 2 (*n* = 100)	Group 3 (*n* = 100)	*F*/*χ*^2^ value	*P* value
Sex (male)	50 (50.00)	51 (51.00)	55 (55.00)	0.561	0.755
Age (years)	48.44 ± 7.43	49.44 ± 6.88	49.02 ± 7.86	0.460	0.632
Heart rate (beats/min)	62.40 ± 9.30	64.32 ± 9.50	64.50 ± 9.42	1.531	0.218
Clinical symptoms					
Chest pain	7 (7.00)	5 (5.00)	9 (9.00)	1.229	0.541
Chest tightness	8 (8.00)	9 (9.00)	6 (6.00)	0.659	0.719
Precordial discomfort	4 (4.00)	2 (2.00)	3 (3.00)	0.687	0.709
Effort angina	3 (3.00)	2 (2.00)	2 (2.00)	0.293	0.864
Past medical history					
Myocardial infarction	2 (2.00)	1 (1.00)	1 (1.00)	0.507	0.776
Hypertension	10 (10.00)	12 (12.00)	14 (14.00)	0.758	0.685
Diabetes mellitus	7 (7.00)	5 (5.00)	8 (8.00)	0.750	0.687

**Table 2:** Comparison of primary puncture success rate, injection success rate, and contrast leakage rate among the three groups of patients (*n*, %).

Group	Number of cases	Primary puncture success	Injection success	Contrast leakage
Group 1	100	95 (95.00)	98 (98.00)	1 (1.00)
Group 2	100	96 (96.00)	99 (99.00)	0 (0.00)
Group 3	100	92 (92.00)	98 (98.00)	3 (3.00)
*F*/*χ*^2^ value	—	1.621	0.407	3.547
*P* value	—	0.445	0.816	0.170

**Table 3:** Comparison of subjective ratings of image quality among the three groups of patients (*n*, %).

Group	Number of cases	Good quality	Good	Barely diagnostic	Unable to assess/fail
Group 1	100	52, (52.00)	41, (41.00)	6, (6.00)	1, (1.00)
Group 2	100	60, (60.00)	34, (34.00)	6, (6.00)	0, (0.00)
Group 3	100	48, (48.00)	42, (42.00)	8, (8.00)	2, (2.00)
*F*/*χ*^2^ value	—	3.000	1.597	0.429	2.020
*P* value	—	0.223	0.450	0.807	0.364

## Data Availability

Data for this experiment are available upon reasonable request to the authors.
